# Effect of Load Carriage Lifestyle on Kinematics and Kinetics of Gait

**DOI:** 10.1155/2023/8022635

**Published:** 2023-02-08

**Authors:** Hsin-Huan Wang, Wei-Chi Tsai, Chi-Yao Chang, Min-Hao Hung, Jui-Hung Tu, Ti Wu, Chia-Hsiang Chen

**Affiliations:** ^1^Graduate Institute of Sports Science, National Taiwan Sport University, Taoyuan, Taiwan; ^2^Rehabilitation Department, Kaohsiung Armed Forces General Hospital Zuoying Branch, Kaohsiung, Taiwan; ^3^Department of Physical Education and Sport Sciences, National Taiwan Normal University, Taipei, Taiwan; ^4^General Education Center, National Penghu University of Science and Technology, Penghu, Taiwan; ^5^Office of Physical Education, National Chin-Yi University of Technology, Taichung, Taiwan; ^6^Department of Physical Education, National Pingtung University, Pingtung, Taiwan; ^7^Office of Physical Education, National Pingtung University of Science and Technology, Pingtung, Taiwan

## Abstract

Backpacks are commonly worn by many people for multiple purposes. This study investigated the effects of habitual wearing of backpacks on lower limb kinematics and kinetics. Fourteen participants were recruited for analysis. All participants performed four randomly assigned scenarios, including running and walking at speeds of 3.5 and 1.5 m/s, respectively, with and without load carriage. The motion analysis system and force plate were used to investigate the lower limb kinematics and kinetics. A paired sample *t*-test was performed for statistical measurement with a significance level of *α* = .05. The results indicated that active force, breaking force, impact peak, loading rate, active peak, maximum braking, hip flexion, and hip range of motion were substantially higher under load carriage conditions than under walking condition, however, time to peak was lower. Conversely, during load carriage running, active force, braking impulse, time to peak, ankle plantarflexion, and ankle range of motion were all higher than those during running. Carrying a backpack weighing 10% of the body weight induced different foot strike patterns at both speeds; during load carriage walking, the hip tended to flex more; whereas, during load carriage running, the ankle tended to flex more. In conclusion, human body seems to adopt different gait strategies during load carriage walking and running. That is, the hip strategy is used during walking, while the ankle strategy is used during running.

## 1. Introduction

Wearing backpacks can alter gait and posture, resulting in musculoskeletal injuries of the lower extremities [1]. Previous studies showed that load carriage affects walking posture and gait and may even cause trunk bending and spinal asymmetry [2, 3], leading to an increased incidence of lower extremity injuries, and even back pain [4]. Therefore, experts have suggested that the backpacks worn by elementary and growing students should not be too heavy [5], with one study stating that it should not exceed 15% of the body weight [6]. The habitual use of backpacks has become fairly common in the daily life of people of many professions, including office workers, students, and the elderly, all of whom can be seen walking or running with a backpack. However, altering gait speed when carrying a load carriage of 10% of body weight may increase lower limb loadings.

Lower extremity injuries can easily occur if the vertical reaction force generated by the ground during walking or running is too high. In general, ground reaction forces generated during walking and running can be 3.5–6 times higher than the body weight, with a faster speed resulting in a higher vertical reaction force [7]. Furthermore, heel contact during fast walking increases musculoskeletal load [8]. Gait speed can affect ground reaction force; hence, it can increase impact force [9], which can result in an increased body burden [10]. All steps involved in lower extremity landing may represent a risk of injury [11]. Different studies have reported varying numbers of basic steps per day for adults, with the average being ∼5,000 steps per day [12]. Whether it is daily walking or running, overuse of the lower extremities is a major cause of injury [13]; therefore, it is important to reduce the risk of overuse injuries. Thus, backpack-loaded walking and running in daily life may indirectly increase the risk of lower extremity injuries. Most studies regarding load carriage have investigated military personnel and children [14, 15], the majority of whom were Caucasians, while fewer studies have investigated Asians. Due to the smaller landscape in many Asian countries, people's lifestyles and gait features may differ from those who live in more spacious regions. This potential difference makes the results of this study quite interesting.

In this context, herein, this study investigated the effect of backpack weight on lower extremity kinetics and kinematics during daily walking and running and proposed two hypotheses: (1) increasing the load carriage affects lower extremity kinetics and kinematics and (2) increasing the gait speed affects lower extremity kinetics and kinematics.

## 2. Methods

### 2.1. Participants

This study recruited 14 young Asian adults who exercise regularly (age: 21.9 ± 1.8 years; height: 161.6 ± 6.1 cm; weight: 51.6 ± 8.3 kg; ten females, four males). None of the participants had any lower extremity nerve, muscle, bone, tendon, or ligament injury, nor any history of cardiovascular problems within the 6 months prior to study initiation. Furthermore, all participants understood the experimental content, procedures, and precautions and were interested in the study before conducting the experiment. This study was approved by the Kaohsiung Armed Forces General Hospital Institutional Review Board (KAFGHIRB 110-012).

### 2.2. Instrumentation

All tests were conducted in an indoor sports biomechanical laboratory. Four dynamic high-speed cameras (Motion Analysis Corporation, Santa Rosa, CA, USA) were used to obtain kinematics data at a capture frequency of 200 Hz. These cameras were set up on a 20 m long runway allowing sufficient distance for acceleration and deceleration. The error value of all cameras was estimated to be <5 mm after calibration [16].

Regarding kinetics data, an AMTI force plate (Advanced Mechanical Technology Inc., Watertown, MA, USA) was used to obtain ground reaction force data at a capture frequency of 1,000 Hz; the force plate was placed 10 m from the starting point on the runway and was aligned with the laboratory floor. The camera and force plate were synchronized using the cortex motion analysis system. The participants started walking/running at 0 m on the runway and stopped at 20 m, i.e., at the end of the runway. They were instructed to step on the force plate for data collection during the walking and running tests.

A self-made-weighted backpack was used in this study (length: 39 cm, width: 24 cm, forth-rear width: 12 cm; Decathlon Groupe, QUECHUA, France), and a weight plate was put inside the backpack, with the weight varying according to the test weight of the participants. The shoulder straps were adjusted so that the center of gravity (lower end of the backpack) was positioned just above the posterior superior iliac spine. The plate was fixed inside the backpack to avoid shaking during the test. Moreover, all participants wore the same model of casual shoes (US6, US8, and US10; 600 g) to reduce the error caused by different shoe models.

### 2.3. Experimental Design

Past studies indicated that carrying a backpack weighing more than 10%–15% of body weight increased the head and trunk forward lean, while a backpack weighing 10% of body weight had no effect on trunk posture [17]. Therefore, experts suggest that backpack weight should not exceed 10% of body weight [18]. A previous study defined 1.5–3.0 m/s as walking speed and 3.5–6.0 m/s as jogging speed [19]. As such, this study used 10% of body weight as the load carriage weight for this study. In addition, simulated walking and running gait speeds used in this study were 1.5 and 3.5 m/s, respectively.

To monitor the anatomical positions of each of the limbs during gait, reflective spheres were stuck according to the Helen Hayes model [20], with a total of 31 markers on the head, upper extremities, pelvis, lower extremities, and feet. To define the model, spheres were adhered to the forehead, top, and back of the head; spheres on the upper limbs were placed on the acromion, lateral elbow, and midpoint of the wrist; those on the pelvis were placed on the anterior and posterior superior iliac spines and the caudal spine; those on the lower limbs were placed on the inner and outer sides of the ankle bone; and those on the feet were placed on the heel bone and midpoint of the first and second metatarsals. Moreover, six markers were added to assist in segment tracing; one marker each was stuck on both arms, thighs, and calves (Figure 1). At least three reflective markers were required for each segment to construct the joint center and define the anatomical position of the limbs in the coordinate system [21].

### 2.4. Procedures

The experimental procedures and actions were explained before conducting the tests, and the participants were familiarized with the procedures. For the test, participants wore their own sports clothing, with the experimental casual shoes and weighted backpack, and reflective spheres were stuck on their whole body for the formal testing.

Before starting the experiment, participants were briefed about the study and protocol, and then changed to clothing and sneakers suitable for exercise. Afterward, participants wore the experimental backpack, and the practitioner positioned the reflective markers on them.

The participants performed four test scenarios in a randomized balanced order. The walking and running tests were conducted both with and without load carriage, with four scenarios in total: walking test without load, running test without load, walking test with load, and running test with load. Each scenario was initiated with a verbal reminder to be prepared, and three acquisitions were made. To be deemed successful, each scenario required that the participant stepped their right foot fully onto the force plate at the targeted speed. The runway was a 20 m-leveled surface with the force plate situated in the middle. A 5 min resting period was ensured between the scenarios to prevent lower extremity muscle fatigue affecting the results.

### 2.5. Data Analysis

The study implemented Cortex motion analysis system, which was synchronized with high-speed cameras and a three degrees of freedom force plate to obtain kinematic and kinetic gait data. The kinematic parameters investigated in this study include hip flexion, hip extension, hip range of motion (ROM), knee flexion, knee extension, knee ROM, ankle dorsiflexion, ankle plantarflexion, and ankle ROM. The kinematic signal of the Cortex motion analysis system was smoothed with a Butterworth 4th-order low-pass filter at 6 Hz [22]. The signal of the force plate was processed in the same manner as that of the kinematic signal. Afterward, the kinetic signal was calculated in the LabVIEW (National Instruments, Austin, TX) to obtain the active force, braking force, active impulse, braking impulse, impact peak, time to impact peak, loading rate, active peak, and maximum breaking. These kinetic parameters were normalized and expressed as Newton's per unit body mass (N BM-1), allowing direct comparison between participants [23]. Only the data of the right leg were included.

### 2.6. Statistical Analysis

In this study, the IBM SPSS software (SPSS Inc., Chicago, USA) was adopted for the statistical analysis. Paired sample *t*-test was performed to analyze the differences in running and walking with and without carrying load carriage system. The significance level was defined at *α* = 0.05. In addition, the Shapiro–Wilk and Levene's homogeneity tests were performed to assess normal distribution. The results indicated that the data were normally distributed. Furthermore, to interpret the resulting number, effect sizes were calculated by the commonly used general guide developed by Cohen [24], in which scores <0.1 = trivial effect, 0.1–0.3 = small effect, 0.3–0.5 = moderate effect, and >0.5 = large effect.

## 3. Results

### 3.1. Kinetic Parameters

Table 1 shows the kinetic parameters of the walking and running tests with and without load carriage. The results showed that during load carriage walking, the active force, braking force, impact peak, time to impact peak, loading rate, active peak, and maximum breaking were all higher than those during walking without a load carriage. During load carriage running, the active force, braking impulse, and time to impact peak were all higher than those during running without a load carriage (Figure 2).

### 3.2. Kinematic Parameters

Table 2 shows the kinematic parameters of the walking and running tests with and without load carriage. During load carriage walking, hip flexion and hip ROM were significantly larger than that during walking without load carriage (Figure 3). Conversely, during load carriage running, ankle plantar flexion and ankle ROM were all higher than those during running without load carriage (Figure 4).

## 4. Discussion

Overall, the findings of this study indicate that the braking force and loading rate were greater and the impact time was lower during walking with load carriage than those without. Furthermore, hip flexion and ROM were greater with load carriage, while ankle dorsiflexion and ROM were greater during running than during walking. All of these results are consistent with the study hypotheses.

The kinetic results demonstrated that the active force and braking force increased during load carriage walking, whereas only the active force increased during the load carriage running scenario. These results agree with those of a previous study that showed that load carriage of 25.6 kg was advantageous to the front/back system propulsion [25]. In this study, the load carried was determined as 10% of body weight, and the final weight, therefore, differed between participants (∼4.3–5.9 kg). Nevertheless, the weight carried by all participants was considerably lighter than previously reported (25.6 kg). Thus, the results indicate that even carrying a lighter weight can elicit the same propulsive effect previously shown by Lloyd and Cooke [25]. Conversely, findings of this study indicated that both load carriages are walking and running increased impact force, which has previously been reported in individuals carrying 6.5%–27.2% body weight, as well as in another study in which the participants carried an excessive 32 kg during walking [26, 27]. Based on our findings, as well as several other reports, it is certain that carrying a backpack of 10% of body weight will increase impact force, thereby increasing the loading rate. This study specifically examined the kinetic effects of walking and running with a loaded backpack. It was found that load carriage walking and running with 10% of body weight would alter lower limb kinetics.

In addition to kinetics, our study observed that load carriage walking increased hip flexion angle, this phenomenon has also been observed in other studies which adopted a load carriage weight of less than 20 kg [28, 29]. These previous findings indicate that carrying lighter weights may also affect hip joint angle. To be more specific, higher stability can be achieved by increasing hip flexion angle [30], which coincided with our finding that an increase in hip flexion angle has also been found when carrying a lighter load carriage weight.

Another interesting finding in this study was that ankle plantarflexion, and ankle ROM increased during load carriage running, which is corroborated by the similar results found in several previous studies [31, 32]. Although load carriage activity affects ankle kinematics, one study previously reported that the ankle plays an important role when the load carried is greater than 30% of body weight [33]. In addition to load carriage, it has been shown that moderate ankle joint motion is important for daily activities [34]. Finally, although increasing the load changes the kinematic parameters of the hip, knee, and ankle joints [35], our study showed that load carriage walking with relatively low weight (10% of body weight) did not result in alterations in the knee joint angles compared to normal walking, thus, during load carriage walking and running, the lower extremity adopts a different gait strategy.

Furthermore, it has been reported that the knee joint angle tends to flex more when carrying loads of more than 10 kg [36], which contradicts our findings. According to past studies, hip, knee, and ankle angles tend to increase at a higher exercise intensity [37–39]. The phenomenon has also been found in the present study, where hip and ankle joint angles increased during load carriage activity with 10% of body weight. However, knee joint angles did not differ under this condition. In light of our findings, load carriage of 10% of body weight is more demanding for the hip and ankle but not for the knee, which may not lead to a higher risk of knee injury.

This study has several crucial findings. First, despite the increasing impact force and loading rate, load carriage of 10% of body weight improves braking force, thereby improving the effective propulsion of the front/back system. Second, the health condition of the ankle should be of concern, especially when carrying a backpack on a daily basis, since the ankle can become a risk factor that affects the health condition of the lower extremity regardless of the weight carried. In addition, hip joint plays an important role on providing stability during load carriage activity; therefore, it is crucial to strengthen the muscle around the hip.

Nevertheless, this study has several limitations that should be mentioned. First, the weights tested in this study were limited to 10% of body weight; therefore, the results of this study may not be generalizable to heavier weights. Another limitation was the backpack type. Only the two-strapped backpack was used in this study, other types, such as one-strap side backpacks and one-strap cross-body bags, may have different effects. Furthermore, there are numerous available designs of the commercial two-strapped backpack; however, only one model was used in this study in order to reduce the discrepancy; as such, the results may be limited to similar backpack designs and functions. Furthermore, this study only included Asians; therefore, the results may not represent the effects in different ethnicities.

## 5. Conclusion

The findings of this study indicate that even carrying a lighter weight (10% of body weight) can significantly alter lower limb kinetics and kinematics. More specifically, load carriage walking and running induce different kinetic and kinematic effects; the human body tends to adopt a more flexed hip angle during load carriage walking, whereas a greater ankle ROM is observed during load carriage running. As a result, human body adopts different gait strategies during load carriage activities; the hip strategy is used during walking, and the ankle strategy is used during running. These results indicate that running should be avoided when carrying a backpack of 10% of body weight in order to reduce loading on the ankles.

## Figures and Tables

**Figure 1:** Load carriage conditions.

**Figure 2:** Gait raw data obtained from the force plate for with load carriage and without load carriage. The *x*-axis shows the normalized gait cycle in percentage.

**Figure 3:** Raw data of the hip, knee, ankle joint angles during walking with and without load carriage. The *x*-axis shows the normalized gait cycle in percentage.  ^*∗*^Indicates a significant difference between with and without load carriage (*p* < .05).

**Figure 4:** Raw data of the hip, knee, ankle joint angles during running with and without load carriage. The *x*-axis shows the normalized gait cycle in percentage.  ^*∗*^Indicates significant difference between with and without load carriage (*p* < .05).

**Table 1:** Descriptive statistics and *p*-values for gait kinetic parameters with and without load carriage.

Kinetic (mean ± SD)								
	Walk		Running		Walk		Running	
	Without load	With load	Without load	With load	*p*	ES	*p*	ES
Active force (%BW)	19.26 ± 2.36	22.53 ± 3.61	22.61 ± 6.13	29.13 ± 8.16	≤.001^*∗*^	1.19	.012^*∗*^	0.82
Braking force (%BW)	−22.27 ± 3.33	−25.64 ± 3.54	−22.97 ± 3.84	−22.98 ± 4.36	.004^*∗*^	0.89	.918	0.04
Active impulse (N × S)	33.36 ± 7.38	29.22 ± 12.67	22.96 ± 2.76	22.32 ± 7.19	.322	0.40	.787	0.12
Braking impulse (N × S)	−33.03 ± 8.40	−29.89 ± 14.49	−14.32 ± 3.11	−18.83 ± 6.29	.437	0.26	.007^*∗*^	0.91
Impact peak (%BW)	111.49 ± 16.78	119.52 ± 8.41	193.42 ± 30.71	189.45 ± 32.92	.010^*∗*^	0.34	.965	0.01
Time to impact peak (S)	0.37 ± 0.07	0.29 ± 0.08	0.10 ± 0.02	0.11 ± 0.03	.005^*∗*^	1.06	.003^*∗*^	0.39
Loading rate (%BW/S)	275.16 ± 83.03	474.89 ± 210.32	1876.75 ± 481.14	1807.57 ± 592.79	.005^*∗*^	1.25	.366	0.13
Active peak (%BW)	102.92 ± 3.57	113.15 ± 5.68	173.92 ± 21.07	178.11 ± 24.57	≤.001^*∗*^	0.37	.205	0.10
Max braking (%BW)	114.58 ± 13.49	123.94 ± 9.71	243.04 ± 35.70	240.49 ± 24.09	≤.001^*∗*^	0.38	.948	0.01

Note: Values are presented as the mean ± SD.  ^*∗*^Indicates significant difference between with and without load carriage (*p* < .05).

**Table 2:** Descriptive statistics and *p*-values for joint kinematics with and without load carriage.

Kinematics (mean ± SD)								
	Walk		Running		Walk		Running	
	Without load	With load	Without load	With load	*p*	ES	*p*	ES
Hip flexion (°)	37.29 ± 5.99	40.56 ± 7.92	44.38 ± 6.91	42.53 ± 9.81	.043^*∗*^	0.47	.502	0.22
Hip extension (°)	−3.67 ± 1.71	−2.73 ± 6.01	3.37 ± 4.59	2.34 ± 7.90	.152	0.16	.686	0.16
Hip ROM (°)	40.96 ± 6.58	43.29 ± 5.99	41.01 ± 7.55	40.19 ± 11.94	.017^*∗*^	0.37	.845	0.10
Knee flexion (°)	6.82 ± 2.92	9.94 ± 5.14	21.48 ± 6.71	20.75 ± 5.29	.086	0.75	.075	0.12
Knee extension (°)	71.09 ± 4.08	68.54 ± 5.11	88.68 ± 11.50	87.52 ± 10.51	.075	0.55	.739	0.11
Knee ROM (°)	64.27 ± 5.58	58.60 ± 8.71	67.21 ± 13.65	66.77 ± 14.60	.065	0.78	.915	0.03
Ankle dorsiflexion (°)	4.22 ± 2.99	3.36 ± 7.17	10.38 ± 7.83	12.08 ± 6.55	.623	0.16	.563	0.24
Ankle plantarflexion (°)	−24.87 ± 7.14	−25.62 ± 2.49	−18.13 ± 8.77	−26.05 ± 4.34	.741	0.14	.039^*∗*^	1.15
Ankle ROM (°)	29.09 ± 7.64	28.99 ± 8.58	28.51 ± 10.67	38.14 ± 7.69	.959	0.01	.046^*∗*^	1.04

Note: Values are presented as the mean ± SD.  ^*∗*^Indicates significant difference between with and without load carriage (*p* < .05).

## Data Availability

The data used to support the findings of this study are included in the article. Please contact the relevant author if you would like to acquire the numerical dataset used to conduct the research described in the paper.
